# Comparison of diagnostic accuracy of Midkine and AFP for detecting hepatocellular carcinoma: a systematic review and meta-analysis

**DOI:** 10.1042/BSR20192424

**Published:** 2020-03-20

**Authors:** Qingqing Lu, Jie Li, Hui Cao, Chenlu Lv, Xiaolin Wang, Shiqiong Cao

**Affiliations:** Division of Gastroenterology, Liyuan Hospital, Tongji Medical College, Huazhong University of Science and Technology, No. 39, Yanhu Avenue, Wuhan, Hubei, China

**Keywords:** AFP, diagnosis, HCC, MDK, meta analysis

## Abstract

**Objective:** Midkine (MDK) has been proposed as one of the most promising markers for hepatocellular carcinoma (HCC). This meta-analysis was conducted to compare the diagnostic accuracy of MDK and α-fetoprotein (AFP) for HCC.

**Methods:** We systematically searched PubMed/MEDLINE, Ovid/EMBASE, and the Cochrane Library for all relevant studies up to 18 May 2019. The Revised Quality Assessment for Studies of Diagnostic Accuracy tool (QUADAS-2) was used to assess the methodological quality of the included studies. The sensitivity, specificity, and the area under the curve (AUC) of MDK and AFP for detecting HCC were pooled using random-effects model.

**Results:** Seventeen studies from five articles with a total of 1122 HCC patients and 2483 controls were included. The summary estimates using MDK and AFP for detecting HCC were as follows: sensitivity, 85 vs 52%, specificity, 82 vs 94%, and AUC, 0.90 vs 0.83. The summary estimates using MDK and AFP for detecting hepatitis virus-related HCC as follows: sensitivity, 93 vs 74%, specificity, 85 vs 97%, and AUC, 0.95 vs 0.97. The summary estimates using MDK and AFP for detecting early-stage HCC were as follows: sensitivity, 83.5 vs 44.4%, specificity, 81.7 vs 84.8%, and AUC, 0.87 vs 0.52. The summary estimates using MDK for detecting AFP-negative HCC as follows: sensitivity, 88.5%, specificity, 83.9%, and AUC, 0.91.

**Conclusion:** MDK is more accurate than AFP in diagnosing HCC, especially for early-stage HCC and AFP-negative HCC. Both MDK and AFP had excellent diagnostic performance for hepatitis virus-related HCC.

## Introduction

Hepatocellular carcinoma (HCC), one of the most prevalent primary malignant tumors, has been a main cause of cancer deaths all over the world with rising incidence rate and mortality [1]. The latest study shows there were 841080 new cases of liver cancer worldwide in 2018 [2]. In addition, HCC is often correlated with poor prognosis due to the lack of sensitive early detection methods and the limitation of effective treatment options [3], with a 5-year survival rate of less than 5% [4], which makes it a tremendous challenge for public health. In Asia and Africa, especially China and Egypt, this challenge is more severe due to the high incidence of viral hepatitis and cirrhosis [5,6]. To improve the prognosis of liver cancer, surveillance guidelines for the early diagnosis of HCC have been proposed [7–9].

Serum α-fetoprotein (AFP), is currently recommended in guidelines, has been used widely in routine practice. Nevertheless, its diagnostic performance is suboptimal [10]. In addition, as many as 40% of HCC patients has normal AFP levels, especially for early HCC [11]. Meanwhile, elevated AFP levels can also be detected in some patients with chronic hepatitis and liver cirrhosis [12,13]. Therefore, an array of alternative markers is urgently need for the diagnosis of HCC at early stage.

Midkine (MDK) is a heparin-binding growth factor with a molecular weight of 13 kDa, strongly expressed at an early stage of differentiation during embryogenesis [14]. However, for normal adults the expression of MDK is present at low levels or undetectable [15]. In recent years, MDK has attracted the attention of many researchers because of its important role in tumor-related activities such as anti-apoptosis, proliferation, transformation, and migration of various tumors including HCC [16]. It has been proposed as one of the most promising markers for HCC. There have been studies estimating the diagnostic performance of serum MDK for predicting HCC [16–20], but the results are inconsistent, especially when compared with AFP. To resolve this controversy, we conducted this meta-analysis to evaluate the diagnostic efficacy of MDK in HCC and compared it with AFP.

## Materials and methods

### Literature search strategy

The PubMed/MEDLINE, Ovid/EMBASE, and the Cochrane Library were searched systematically for all eligible studies published until 18 May 2019 using the following search terms: (‘Midkine’ or ‘MDK’ or ‘MK’) and (‘Carcinoma, Hepatocellular’ or ‘Liver Neoplasms’ or ‘hepatocarcinoma*’ or ‘hepatoma*’or ‘HCC’ or ((‘Hepatocellular’ or ‘liver cell’ or ‘hepatic cell’ or ‘liver’) and (‘carcinoma*’or ‘tumor’))). In addition, the list of references was manually searched.

### Inclusion and exclusion criteria

Only articles that met all the following criteria were included in this meta-analysis: (i) studies that directly compared the predictive performance of MDK with AFP for HCC in the same patients; (ii) the studies included sufficient data to construct 2 × 2 table that consisted of the true positives (TPs), false positives (FPs), true negatives (TNs), and false negatives (FNs); (iii) the diagnosis of HCC was confirmed based on histology or the appropriate imaging characteristics as defined by accepted guidelines; (iv) serological samples were collected to measure the levels of MDK and AFP. The studies that contain any of the following criteria will be excluded: (i) irrelevant topics; (ii) conference abstracts, letters, comments, editorials, guidelines, reviews, case reports; (iii) animal or cellular experiments. These studies contained in this meta-analysis were assessed by two investigators independently.

### Definition of HCC, hepatitis virus-related HCC, early-stage HCC, and AFP- negative HCC

HCC was diagnosed based on histology or the appropriate imaging characteristics as defined by accepted guidelines [21]. Hepatitis virus-related HCC was defined based on a background of chronic hepatitis and corresponding cirrhosis. Early-stage HCC and AFP-negative HCC were defined as BCLC 0-A (Barcelona Clinic Liver Cancer) and AFP less than 20 ng/ml, respectively.

### Data extraction and quality assessment

We developed a data extraction sheet, pilot-tested it on five randomly selected included studies, and refined it accordingly. One review author extracted the data from included studies and the second author checked the extracted data. These data including basic characteristics of each included study (authors, year of publication, region, etiology and characteristics of HCC, number of patients and controls, assay type of MDK and AFP) and the performance indices of MDK and AFP (cut-off values, TP, FP, FN, TN). The disagreements were resolved by discussion between the two review authors; if no agreement could be reached, it was planned a third author would decide. The methodological quality of the included studies was assessed according to the Quality Assessment of Diagnostic Accuracy Studies (QUADAS) [22].

### Data synthesis and analysis

Statistical analysis was performed by Stata version 12.0 (STATA Corp, MIDAS module), and Meta-Disc version 1.4 (XI Cochrane Colloquium, Barcelona, Spain). The sensitivity (Se), specificity (Sp), positive likelihood ratio (PLR), negative likelihood ratio (NLR), and diagnostic odds ratio (DOR) were pooled to evaluate the diagnostic accuracy of MDK and AFP for HCC. Meanwhile, the summary receiver operating characteristic (SROC) curve was drawn, and the corresponding area under the curve (AUC) was obtained. A diagnostic tool is defined as perfect if AUC is 1.00, excellent if the AUC is greater than 0.90, good if it is greater than 0.80, moderate if it is less than 0.80 [23]. The methodological quality of the included studies was assessed using Review Manager 5.3 (Cochrane Collaboration, Copenhagen, Denmark).

### Assessment of heterogeneity and publication bias

Heterogeneity is used to describe the degree of variation in effect sizes in a series of studies. Q statistic of χ^2^ value test and inconsistency index *I^2^* were used to evaluate the heterogeneity between studies. The *I^2^* > 50% or *I^2^* > 25% with a *P*-value < 0.10 indicated that the heterogeneity was substantial [24]. Meta-regression analysis was used to identify potential sources of the heterogeneity between the included studies [25]. In addition, Spearman’s correlation coefficient wais utilized to verify the possibility of a threshold effect. A strong positive correlation would prove the existence of threshold effect. Publication bias refers to the reluctance of researchers, journal editors, and study sponsors to publish studies with small sample size or no statistical significance. Therefore, it has become an important task for meta-analysis to examine whether publication bias exists on results [26]. Deeks’ funnel plot was used to detect publication bias. Generally, two-sided *P*<0.05 was considered to be statistically significant.

## Results

### Basic characteristics of the retrieved studies

A total of 374 records were retrieved using our search strategy, of which 184 were repeated. After reviewing the titles and abstracts, 177 records were removed because they were either only abstracts or reviews, either animal experiments or not relevant to the current analysis. Next, we further evaluated the remaining 13 articles. Of these, eight articles were excluded for the following reasons: two items were not relevant to the topic, two items were excluded due to lack of serum samples, and four items did not provide enough data to construct 2 × 2 table for diagnostic performance. Finally, five eligible articles including 17 studies were enrolled in this meta-analysis [16–20]. A total of 3605 described subjects participated in the current analysis, including 1122 patients and 2483 controls. Flow diagram of study selection is shown in Figure 1. All the studies were published between 2013 and 2018. Most of the included studies were from China (five studies), Egypt (seven studies), and Australia (five studies). Among them, five studies and four studies independently assessed the diagnostic accuracy of MDK and AFP for hepatitis virus-related HCC and early-stage HCC. In addition, three studies evaluated the predictive performance of MDK for AFP-negative HCC. ELISA was selected by all studies to test MDK. The assay methods of AFP were inconsistent. According to whether the serum AFP was positive or not, we divided 17 studies into two groups. The detailed characteristics of each studies in two groups are listed in Tables 1 and 2.

**Figure 1:** Flow diagram of study selection *From:* Moher D., Liberati A., Tetzlaff J., Altman D.G. and The PRISMA Group (2009). *P*referred *R*eporting *I*tems for *S*ystematic Reviews and *M*eta-*A*nalyses: the PRISMA Statement. *PLoS Med.* 6(6): e1000097, doi:10.1371/journal.pmed1000097. For more information, visit www.prisma-statement.org.

**Table 1:** Characteristics of the included studies in group1

Author	Year	Region	Patients	Controls	MDK		AFP	
					Assay type	Cutoff (ng/ml)	Assay type	Cutoff (ng/ml)
Mashaly et al. [16]	2018	Egypt	HCC	A	ELISA	1.683	ELISA	200
Hodeib et al. [17]	2017	Egypt	HV-HCC	D	ELISA	0.650	EIA	80
Vongsuvanh et al. [18]	2016	Australia	HCC	A+E	ELISA	0.440	CLIA	20
Vongsuvanh et al. [18]	2016	Australia	Early HCC	A+E	ELISA	0.440	CLIA	20
Vongsuvanh et al. [18]	2016	Australia	HV-HCC	A	ELISA	0.440	CLIA	20
Vongsuvanh et al. [18]	2016	Australia	HV-HCC	A+F	ELISA	0.440	CLIA	20
Vongsuvanh et al. [18]	2016	Australia	HCC	A	ELISA	0.440	CLIA	20
Shaheen et al. [19]	2015	Egypt	HV-HCC	A	ELISA	0.387	CLIA	88.5
Shaheen et al. [19]	2015	Egypt	HV-HCC	D	ELISA	0.387	CLIA	88.5
Shaheen et al. [19]	2015	Egypt	Early HCC	A	ELISA	0.387	CLIA	88.5
Zhu et al. [20]	2013	China	HCC	A+B+C+D	ELISA	0.654	NK	20
Zhu et al. [20]	2013	China	Early HCC	A	ELISA	0.654	NK	20
Zhu et al. [20]	2013	China	HCC	A+B+C+D	ELISA	0.654	NK	20
Zhu et al. [20]	2013	China	Early HCC	A+B+C+D	ELISA	0.654	NK	20

*Group 1*: Studies assessed the diagnostic accuracy of MDK and AFP for HCC.

Abbreviations: A, cirrhosis; B, hepatic benign tumor; C, other digestive cancer patients; CLIA, chemiluminescence immunoassay; D, healthy people; E, chronic liver disease; Early HCC, early-stage HCC; EIA, enzyme immunometric assayELISA, enzyme-linked immunosorbent assay; F, chronic hepatitis B; HV-HCC, hepatitis virus-related HCC; NK, not known.

**Table 2:** Characteristics of the include studies in group 2

Author	Year	Region	HCC feature	Controls	Assay type	Cutoff (ng/ml)	TP	FP	FN	TN
Mashaly et al. [16]	2018	Egypt	AFP negative	A	ELISA	1.683	17	5	4	26
Shaheen et al. [19]	2016	Egypt	AFP negative	A	ELISA	0.387	14	5	1	25
Zhu et al. [20]	2013	China	AFP negative	A+B+C+D	ELISA	0.654	108	73	13	382

Group 2: Studies assessed the diagnostic accuracy of MDK for AFP- negative HCC. Abbreviations: A, cirrhosis; AFP negative, α-fetoprotein <20 ng/ml; B, hepatic benign tumor; C, other digestive cancer patients; D, healthy people; ELISA, enzyme-linked immunosorbent assay.

QUADAS-2 is used to evaluate the methodological quality of the enrolled studies, and the results are presented in Figure 2. Most of the studies were retrospective, and none indicated that the patient sample was randomized or continuous. As a result, the patient selection items in these studies were labeled ‘unclear’. Only two studies set diagnostic thresholds in advance. Therefore, the conduct or interpretation of the index test in most of the studies were labeled as ‘high risk’. Regarding the reference standard and the flow and timing domain, the studies included in the meta-analysis met the all items and were labeled as ‘low risk’.

**Figure 2:** Methodological quality of included studies according to the revised quality assessment for studies of diagnostic accuracy tool (QUADAS-2) (+, yes; −, no; ?, unclear)

### Diagnostic accuracy of MDK and AFP for HCC

In group 1, 14 studies from five articles [16–20] that directly compared the diagnostic accuracy of MDK with AFP for HCC in the same patients were enrolled. As is shown in Table 3, the pooled sensitivity using MDK (85%) is higher than using AFP (52%) for detecting HCC. However, the pooled specificity of MDK (82%) is inferior to that of AFP (94%). Next, the SROC curves were drawn (Figure 3A,B). The summary AUC values using MDK and AFP for detecting HCC were 0.90 vs 0.83, indicating that MDK is superior to AFP.

**Figure 3:** SROC curve for the diagnostic accuracy of MDK and AFP for HCC (**A,B**) SROC curve for the diagnostic accuracy of MDK (A) and AFP (B) for HCC. Abbreviations: CI, confidence interval; SENS, sensitivity; SPEC, specificity.

**Table 3:** Summary of Se, Sp, PLR, NLR, DOR, and AUC of MDK and AFP for prediction of HCC, hepatitis virus-related HCC, early-stage HCC, and AFP-negative HCC

	Se% [95% CI]	Sp% [95% CI]	PLR [95% CI]	NLR [95% CI]	DOR [95% CI]	AUC [95% CI]
HCC						
MDK	85.0 [78, 90]	82.0 [74,88]	4.7 [3.0,7.4]	0.18 [0.11,0.30]	26 [10, 64]	0.90 [0.87, 0.93]
AFP	52.0 [39,65]	94.0 [87,97]	8.9 [3.9,20.2]	0.51 [0.38,0.68]	17 [7, 47]	0.83 [0.80, 0.86]
Hepatitis virus-related HCC						
MDK	93.0 [72, 99]	85.0 [62, 95]	6.3 [2.0, 20.4]	0.08 [0.02, 0.45]	77 [5, 1215]	0.95 [0.93, 0.97]
AFP	74.0 [41, 92]	97.0 [89, 99]	23.2 [6.5, 83.4]	0.27 [0.10, 0.76]	86 [15, 500]	0.97 [0.94, 0.98]
Early-stage HCC						
MDK	83.5 [78.4, 87.7]	81.7 [78.4, 84.8]	4.28 [1.98, 9.22]	0.217 [0.09, 0.52]	20.76 [4.43, 97.28]	0.89
AFP	44.4 [38.3, 50.6]	84.8 [81.6, 87.5]	3.12 [0.94, 10.37]	0.781 [0.61, 1.00]	3.986 [0.84, 18.87]	0.52
AFP negative HCC						
MDK	88.5 [82.5, 93]	83.9 [81, 87]	5.5 [4.5, 6.8]	0.143 [0.09, 0.22]	40.5 [23.19, 70.76]	0.91

Abbreviation: CI, confidence interval.

### Diagnostic accuracy of MDK and AFP for hepatitis virus-related HCC

In group 1, five studies from three articles [17–19] that directly compared the diagnostic accuracy of MDK with AFP for hepatitis virus-related HCC in the same patients were enrolled. As is shown in Table 3, the pooled sensitivity using MDK (93%) is higher than using AFP (74%) for hepatitis virus-related HCC. However, the pooled specificity of MDK (85%) is inferior to that of AFP (97%). Next, the SROC curves were drawn (Figure 4A,B). The summary AUC values using MDK and AFP for detecting hepatitis virus-related HCC were 0.95 vs 0.97, indicating that AFP is superior to MDK. Both MDK and AFP had excellent diagnostic performance for detecting hepatitis virus-related HCC.

**Figure 4:** SROC curve for the diagnostic of MDK and AFP for hepatitis virus-related HCC (**A,B**) SROC curve for the diagnostic accuracy of MDK (A) and AFP (B) for hepatitis virus-related HCC. Abbreviations: CI, confidence interval; SENS, sensitivity; SPEC, specificity.

### Diagnostic accuracy of MDK and AFP for early-stage HCC

In group 1, four studies from three articles [18–20] that directly compared the diagnostic accuracy of MDK with AFP for early-stage HCC in the same patients were enrolled. As is shown in Table 3, the pooled sensitivity using MDK (83.5%) is higher than using AFP (44.4%) for early-stage HCC. However, the pooled specificity of MDK (81.7%) is inferior to that of AFP (84.8%). Next, the summary AUC values using MDK and AFP for detecting early-stage HCC were pooled with AUC values 0.87 vs 0.52, indicating that MDK is superior to AFP. Serum MDK can be used as a potential marker for early diagnosis of HCC.

### Diagnostic accuracy of MDK for AFP-negative HCC

In group 2, three studies from three articles [16,19,20] that assessed the diagnostic accuracy of MDK for AFP-negative HCC were enrolled. As is shown in Table 3, the summary estimates of sensitivity, specificity, and AUC for MDK in predicting AFP-negative HCC were 88.5, 83.9%, and 0.91, respectively, indicating that serum MDK can be used as a supplementary method for the diagnosis of HCC, especially for AFP-negative HCC.

### Heterogeneity and publication bias

A total of 17 studies were included in this meta-analysis. The forest plots of MDK and AFP are shown in Figure 5A,B, indicating that there was significant heterogeneity among the included studies. In general, threshold effect is one of the most common sources of heterogeneity in diagnostic tests. We identified the threshold effect by Spearman correlation analysis. The results showed that the Spearman’s correlation coefficient of MDK and AFP were 1.00 (*P*=1.00) and 0.361 (*P*=0.204), respectively, indicating no threshold effect. Subsequently, a meta-regression analysis was conducted to explore the potential sources of heterogeneity. As is shown in Table 4, the diagnostic accuracy of MDK for HCC were not affected by sample size, region, published year, etiology of HCC, the composition of the control group and assay type. The diagnostic accuracy of AFP for HCC were not affected by sample size, published year, and etiology of HCC. However, we found that differences in region, assay type, and the composition of the control group had a statistically significant effect on the heterogeneity of AFP in the diagnosis of HCC. Deeks’ funnel plot was constructed to estimate the publication bias. There was no publication bias for MDK and AFP for detecting HCC with *P*=0.81 (Figure 6A) and *P*=0.08 (Figure 6B).

**Figure 5:** Forest plots of MDK and AFP (**A,B**) Forest plots of MDK (A) and AFP (B).

**Table 4:** Meta-regression analyses of potential source of heterogeneity

Variable	MDK		AFP	
	*Coeff*	*P*-value	*Coeff*	*P*-value
Sample size	−0.780	0.6109	−0.003	0.9971
Region	−1.225	0.6038	−4.849	0.0154
Year	−3.599	0.0718	−1.150	0.1976
Etiology of HCC	1.526	0.2328	1.230	0.1328
Control	−1.361	0.2594	−1.522	0.0358
Assay type	-	-	−2.398	0.0483

Abbreviation: Coeff, coefficient.

**Figure 6:** Publication bias of MDK and AFP for the diagnosis of HCC (**A,B**) Deeks’ funnel plot for publication bias on the pooled DOR of MDK (A) and AFP (B) for the diagnosis of HCC.

## Discussion

Due to the lack of accurate early diagnostic methods, HCC has become one of the leading causes of cancer deaths all over the world. Serum AFP is the only diagnostic marker recommended in the Asian guidelines. However, its diagnostic performance is unsatisfactory with low sensitivity and specificity. Over the past decade, advances in genomics, proteomics platforms, and biomarker detection techniques have led to the identification of many new biomarkers to improve the diagnosis of HCC, such as osteopontin (OPN), microRNAs, and MDK [27]. A meta-analysis showed that OPN has a comparable accuracy with AFP for the diagnosis of HCC, but it is limited to diagnosing early HCC [28]. A panel of miRNAs have been identified as promising biomarkers, but the diagnosis of liver cancer using a single miRNA is not reliable enough. Moreover, there is a wide variety of miRNAs, so it is necessary to conduct further studies to determine HCC specific miRNAs [27]. MDK, an emerging serum marker, activates several cell surface receptors to participate in modulating various biological activities and is significantly increased in HCC [29]. It has been proposed as one of the most promising methods for the diagnosis of HCC. However, the results of studies on whether MDK is superior to AFP are inconsistent or even contrary, and most of those studies recruited relatively small size of participants. Therefore, we conducted this meta-analysis which was the first to evaluate the diagnostic efficacy of MDK for HCC and compared it with AFP.

A total of 17 studies from five articles [16–20] were included in this meta-analysis. Among them, 14 studies (group 1) compared the diagnostic efficacy of MDK and AFP for HCC, 5 studies compared the diagnostic accuracy of MDK and AFP for hepatitis virus-related HCC, and 4 studies compared the predictive performance of MDK and AFP for early-stage HCC. As is shown in Table 3, the diagnostic accuracy of MDK is superior to AFP for HCC, especially for early-stage HCC with AUC values were 0.90 vs 0.83 and 0.87 vs 0.52, respectively. The summary AUC values using MDK and AFP for detecting hepatitis virus-related HCC were 0.95 vs 0.97, indicating that AFP is superior to MDK. In addition, the value of MDK in the diagnosis of AFP-negative HCC was assessed. Data from three studies (group 2) were pooled and the results showed that MDK had satisfactory diagnostic efficacy, with an AUC value as high as 0.91. Serum MDK can be used as a supplementary method for the diagnosis of HCC, especially for AFP-negative HCC.

However, there is remarkable heterogeneity between included studies. First, we identified the threshold effect by Spearman correlation analysis. The results showed that the Spearman’s correlation coefficient of MDK and AFP were 1.00 (*P*=1.00) and 0.361 (*P*=0.204), respectively, indicating no threshold effect. Subsequently, a meta-regression analysis was conducted to explore the potential sources of heterogeneity. As is shown in Table 4, the diagnostic accuracy of MDK for HCC were not affected by sample size, region, published year, etiology of HCC, the composition of the control group, and assay type. Meanwhile, the diagnostic accuracy of AFP for HCC were also not affected by sample size, published year, and etiology of HCC. However, we found that differences in region, assay type, and the composition of the control group responsible for the heterogeneity of AFP. Additionally, Deeks’ funnel plot showed that there was no publication bias for MDK and AFP for detecting HCC with *P*=0.81 and *P*=0.08.

There are several strengths to the present meta-analysis. First, it is the first meta-analysis to comprehensively assess the diagnostic performance of serum MDK for HCC, and settle the controversy about whether MDK is superior to AFP. Second, the study design was written in accordance to the Preferred Reporting Items for Systematic Reviews and Meta-Analyses (PRISMA) statement [30]. In addition, studies were selected according to rigorous inclusion and exclusion criteria. However, it has to be noted that there are several limitations in the present study. First, in this meta-analysis, there is significant heterogeneity among the included studies. Although we found that the heterogeneity in AFP group may come from the differences in region, assay type, and the composition of the control group through meta-regression analysis, unfortunately, we failed to find the factors responsible for the existing heterogeneity in MDK group. Second, although the comprehensive literature search has been carried out, the number of relevant studies included in our meta-analysis is still inadequate. All of them came from three countries, China, Egypt, and Australia. The applicability of MDK for the diagnosis of HCC in other countries and regions is unknown. Therefore, before serum MDK can be used as a diagnostic tool for HCC, a large-scale, well-designed, multinational and multicenter clinical study is needed.

## Conclusion

MDK is more accurate than AFP in diagnosing HCC, especially in detecting early-stage HCC and AFP-negative HCC. Both MDK and AFP had excellent diagnostic performance for detecting hepatitis virus-related HCC. Serum MDK may serves as a potential diagnostic marker for HCC and may be used in addition to AFP to increase the sensitivity of HCC detection.

## Abbreviations

AFP: α-fetoprotein
AUC: area under the curve
DOR: diagnostic odds ratio
FN: false negative
FP: false positive
HCC: hepatocellular carcinoma
MDK: Midkine
OPN: osteopontin
QUADAS: Quality Assessment for Studies of Diagnostic Accuracy
SROC: summary receiver operating characteristic
TN: true negative
TP: true positive
